# Dance Movement Recognition Based on Multimodal Environmental Monitoring Data

**DOI:** 10.1155/2022/1568930

**Published:** 2022-07-19

**Authors:** Xiao Lei Liu

**Affiliations:** Music and Dance College of Xinyang Normal University, Xinyang, Henan 464000, China

## Abstract

Fine motion recognition is a challenging topic in computer vision, and it has been a trendy research direction in recent years. This study combines motion recognition technology with dance movements and the problems such as the high complexity of dance movements and fully considers the human body's self-occlusion. The excellent motion recognition content in the dance field was studied and analyzed. A compelling feature extraction method was proposed for the dance video dataset, segmented video, and accumulated edge feature operation. By extracting directional gradient histogram features, a set of directional gradient histogram feature vectors is used to characterize the shape features of the dance video movements. A dance movement recognition method is adopted based on the fusion direction gradient histogram feature, optical flow direction histogram feature, and audio signature feature. Three components are combined for dance movement recognition by a multicore learning method. Experimental results show that the cumulative edge feature algorithm proposed in this study outperforms traditional models in the recognition results of HOG features extracted from images. After adding edge features, the description of the dance movement shape is more effective. The algorithm can guarantee a specific recognition rate of complex dance movements. The results also verify the effectiveness of the movement recognition algorithm in this study for dance movement recognition.

## 1. Introduction

Motion recognition is one of the most popular research directions in the field of computer vision. Its application range covers intelligent human-computer interaction, virtual reality, and motion-aided analysis [1]. Many achievements have been made in the application of motion recognition in virtual reality. However, there is still little research on the combination of motion recognition technology based on video and dance video. Dance movement has many problems, such as high complexity and self-closing. The further development of dance analysis requires video-based motion recognition [2]. The successful application of motion recognition technology in other fields provides a sufficient theoretical basis for its application in dance video motion recognition. In the analysis of dance videos, motion recognition technology reduces the work intensity. It facilitates the retrieval of dance video data, makes the automatic choreography system more efficient, and obtains more colorful results [3].

Multimodal machine learning (mmml) [4] aims to build a model to process and correlate information from various patterns. Multimodal machine learning is divided into representation, translation, alignment, fusion, and colearning. It has vital significance and extraordinary application potential. In nature, every source or presentation of information is called a pattern. Baltrusaitis et al. [5] combined human bone data with a human peripheral contour shape to improve human motion recognition ability. Shahroudy et al. [6] proposed a multimode fusion method based on 3D data and discussed the impact of different fusion methods on recognition accuracy. Ng et al. [7] proposed a new shared specific feature decomposition network based on a depth automatic encoder, which separates the input multimodal signals into a component hierarchy.

Based on the above methods, this study proposes an effective feature extraction method for the dance video dataset. Its main mechanism is to segment the video equally and perform edge feature operations on the segmented video at the same time. The edge features of all video images in each segment are added to one embodiment, and the direction elements of the gradient histogram are extracted. Finally, through the experiment, a set of directional gradient histogram feature vectors *D* is used to characterize the shape features of video dance movements. A dance motion recognition method based on histogram feature, optical flow direction histogram, and audio feature is proposed. This study solves the problem of heterogeneous feature fusion. The multimode environmental monitoring method is adopted to organically integrate three features for dance movement recognition research.

## 2. Multimodal Environmental Monitoring and Identification Mechanism

A local feature is a distinguishable description extracted from the region of interest of the task, as far as the human motion recognition task is concerned [8]. The recognition mode extracts the trajectory of human limbs and the texture of the human body to describe human motion [9].

Researchers widely recognize the application histogram of directional gradient (HOG) feature in visual retrieval tasks. This feature was first proposed by Dalal et al. in 2005 and achieved excellent results in pedestrian detection tasks [10]. The HOG feature representation process includes the following steps: grayscale, image correction, gradient calculation, overlapping fast histogram normalization, and combined histogram block feature. Based on the distribution of edge direction, the HOG feature can better represent the contour of the human body. HOG is not sensitive to the color of light. Compared with the original image, its acquisition process is a dimension reduction operation, which allows the human body to have the following subtle body movements without affecting detection results. Many researchers of human action recognition will also learn from the idea of HOG and add it to the characteristics of human action [11].

Klaser et al. proposed the 3D orientation gradient histogram HOG3D feature for human motion recognition for the first time to solve the problem of insufficient quantization of HOG feature direction [12]. As shown in Figure 1, his main improvement is the dodecahedral representation used for direction quantization and, finally, histogram formation.

Four-dimensional average vector direction histogram (HON4D) is shown. As shown in Figure 2, Oreifei et al. regarded the depth map sequence as a four-dimensional hyperspace, which contains three-dimensional point cloud data and one-dimensional time series, and proposed the feature description of HON4D. This method is similar to HOG3D [13]. First, the average vector of four-dimensional space is obtained, and then, the direction is quantized using a 120 frontal body representation. The calculation of this method is more complicated, which is not suitable for real-time tasks. Besides, the quantization of gradient direction is too complex, and the detailed description of human movement is not strong.

The above researchers put forward new research ideas from the application of the oriented gradient (HOG) feature in visual retrieval tasks and the first proposed 3D-oriented gradient histogram HOG3D feature for human motion recognition. Optical flow direction histogram features and audio features are from the appearance and shape of the dance movements in the video to the movements of the human dance movements, and with the help of audio features, the characteristics of the dance movements are described.

## 3. Dance Movement Recognition Method

Given the specific ability of a single element, this study uses the linear weighted combination method of the multikernel learning method to fuse the HOG feature, optical flow direction histogram feature, and audio feature to complement each other and improve the recognition ability of the classifier [14]. The specific process is to set a set of kernel functions for each component, and each kernel function has a corresponding weight. Finally, multiple kernel functions are combined to form a new kernel function in a linear weighted way [15]. Then, a support vector machine classifier is used for multiclass classification.  Figure 3 shows the fusion process of multicore learning features.

In support vector machines based on multikernel learning, the task of the multikernel learning model training stage is to learn and solve the weight order of each kernel function and the parameters *a* and *b* of the support vector machine classifier. Based on the SimpleMKL algorithm idea introduced by Rakotomamonjy et al. [16], in the previous section, the objective function of the algorithm in this study is defined as

(1) $$\begin{array}{c} \underset{\beta_{g},\beta_{f},\beta_{m},\alpha ,b}{\min}J=\frac{1}{2}\sum_{g=1}^{G}\beta_{g}\alpha^{T}K_{g}\alpha +\frac{1}{2}\sum_{f=1}^{F}\beta_{f}\alpha^{T}K_{f}\alpha +\frac{1}{2}\sum_{m=1}^{M}\beta_{m}\alpha^{T}K_{m}\alpha +C\sum_{i}\xi_{i},\\ \text{s}.\text{t}:y_{i}\left(\sum_{g=1}^{G}\beta_{g}K_{g}\left(x_{i}\right)+\sum_{f=1}^{F}\beta_{f}K_{f}\left(x_{i}\right)+\sum_{m=1}^{M}\beta_{m}K_{m}\left(x_{i}\right)\right)\alpha +y_{i}b\geq 1-\xi_{i}\forall i,\\ \xi_{i}\geq 0,\;\forall i,y_{i}\neq \sum_{g=1}^{G}\beta_{g}+\sum_{f=1}^{F}\beta_{f}+\sum_{m=1}^{M}\beta_{m}=1. \end{array}$$

According to the idea of the implemented algorithm, use the gradient descent algorithm to minimize the objective function of learning and solve the optimal parameters [17]. The specific process is that in each generation selection process, calculate the classifier parameters *a* and *b* by giving the weight order of the kernel function. Then, obtain a new kernel weight order by providing *a* and *b*. Therefore, show the classification function based on a multikernel learning support vector machine as follows [13]

(2) $$\begin{array}{c} y=F\left(x\right)=\left[\sum_{g=1}^{G}\beta_{g}K_{g}\left(x\right)+\sum_{f=1}^{F}\beta_{f}K_{f}\left(x\right)+\sum_{m=1}^{M}\beta_{m}K_{m}\left(x\right)\right]\alpha +b. \end{array}$$

In addition, equation (2) is a binary classification function, and the recognition problem we want to solve in this study is a multicategory classification problem. Therefore, it is necessary to transform the binary classification problem into a multiclassification problem. Divide SVM-based multiclass classification strategies into two types: one versus one and one versus many.

1. One versus one: N class classification problems require N (n-1)/2 classifiers, each of which trains two class samples. When classifying the unknown samples, counter the votes of N categories in all classifiers and the category with the most votes in the category of the location samples.
2. One versus rest: one versus rest strategy for all samples, group the instances of one category into one category, and group the representatives of all remaining types into another category. For N class classification problems, this strategy requires training N classifiers. When training each classifier, assign a class of samples a positive label and give all the harmful brands.

This study chooses the second strategy in classification. Transform the multiclass problems in this study into multiple joint dichotomies. For each category in the dataset, all dance movements in this category are marked as positive and keep other dance movements as unfavorable [18]. The SimpleMKL algorithm trained *P* class SVM classifiers to assume *P* class dance movements. Therefore, the following equation shows the objective function of the multiclass classification.

(3) $$\begin{array}{c} J=\sum_{p=1}^{P}J_{p}\left(\beta_{g},\beta_{f},\beta_{m},\alpha_{p},b_{p}\right). \end{array}$$

In equation (3), *J*_P_ is the machine binary classifier of the *P* support vector. Output the *P* dance movement. A negative sample is a category that is not a *P* dance movement. Finally, the algorithm in this study obtains action categories according to the following formula when conducting multicategory classification:

(4) $$\begin{array}{c} y=\arg\underset{y_{p}}{\max}F_{p}\left(x\right). \end{array}$$

## 4. Dance Movement Recognition and Result Analysis

### 4.1. Dance Dataset

The research on the combination of motion recognition technology and dance has just started. There are still few available dance datasets, including the motion capture dataset of Carnegie Mellon University and the DanceDB dataset of Virtual Reality Laboratory of the University of Cyprus. But the public dataset contains very little dance data—the data used for dance movement recognition research. The FolkDance dataset made by the team laboratory is used in this experiment. The FolkDance dataset is divided into four groups of dances, each of which contains several subdivided dance movements with rich movement categories. Each group of dance movements is relatively complex and challenging.

The motion capture device Vicon is used to collect professional dance movements in the FolkDance dataset. During making the dataset, I designed four groups of FolkDance movements after discussion with dance experts according to the dataset making plan.

The production of FolkDance datasets takes into account the situation of solo dances, regardless of changing stage backgrounds and props. Record 84 dance videos, and set the environment and camera angle in each video as fixed. Set the frame rate of images in the video as 20fps, and the size of each frame is 480 × 360. This dataset contains many dance movements that meet the recognition research requirements in the dance video movement. Use this dataset to verify the effectiveness of the dance movement recognition algorithm proposed in this study. FolkDance dataset mainly includes four groups of dances:

  Two-flower combination with step
  One-flower combination with inside
  Paper towel
  One-flower combination

The specific dance movement classification and sample frames for each group are provided.

#### 4.1.1. Follow Step Double Flower Combination

There are seven dance movements in the combination of double flowers in heel step: double flowers in heel step, small dance on the head, front kick of key position flower, cut flower in a circle, cut flower in the circle from low to high, squat and cross-step, and two drums.  Figure 4 shows the example frames of this combination.

#### 4.1.2. The Combination of Cut and Flower

There are five dance movements in the combination of the inside scene, namely, the kick after the inside location, the cross move, the head move, the pull in the following step, and the cross move.  Figure 5 shows the example frames of this combination.

#### 4.1.3. Towel Flower Combination

Towel flower combination includes eight dance movements: towel flower four drum, point kicking step, head flower cross, forearm flower cover cross, large alternating flower cross, shoulder flower, breaking and winding flower forward and backward, towel flower six drum.

#### 4.1.4. Mosaic Combination

The combination includes eight dance movements: point stand step, press and kick step 1, double hand chip turn simultaneously, double hand chip press and kick step, broken step circle chip left, broken step circle chip right, press and kick step 2, jump, and kick step double hand chip. It notes that there are two pressing back kick movements in this combination. The above two movements are not the same but similar. Here, we mark them by serial number to distinguish them. This combination is shown in Figure 7.

### 4.2. Experimental Environment

The experimental environment used in this study is as follows: CPU: Intel (*R*) Core (TM) 15-4460@3.20GHZ, 8 GB. Operating system used is Ubuntu, 64-bit.

Development environment: MATLAB 2012b, SimpleMKL, OpenCV 2.4.8. SimpleMKL multicore learning open-source library, the implementation of the multicore learning algorithm; OpenCV is an open-source library for computer vision, which is mainly written by C and C++ languages, and can be used across platforms, realizing many commonly used algorithms in computer vision.

### 4.3. Experimental Design

In the specific experimental design of this study, we verify the algorithm and the recognition effect of all single features on two dance datasets [19]. Considering that the FolkDance dataset is divided into four different groups of dances, the recognition effect of the proposed method and single feature is verified in each group.

The experiment extracts three features: histogram feature of direction gradient, straight optical flow direction, square feature, and audio signature feature [4]. For the directional gradient histogram feature, we proposed a method of segmenting the video and performing the operation of cumulative edge features. Considering that the rate of the two datasets is 20*f*_ps_ and the error of the segmented video is about 10 seconds, through the analysis of the dance, the movement difference is relatively small within a second, that is, the dance movement shape changes very little. So, we set the bisection value for each video segment to 10. The divide extraction process of audio signature features into two parts: first, extract the audio stream from the dance video; second, remove the 32-dimensional audio signature features from each frame of the audio stream. The literature constructs audio dictionaries according to the word bag model's ideal for audio signature features and sets the audio dictionary size to 50. The kernel functions used in this study are the Gaussian kernel and histogram cross kernel.

This study refers to the previous research methods of motion recognition multifeature fusion [20], and based on different motion recognition multifeature fusion research methods, the performance of the proposed algorithm is mainly verified from four aspects.

1. Evaluation of different characteristics: this experiment gave the recognition results of a single feature on two dance datasets and the recognition results of the feature fusion method using the multikernel learning method, compared them, and analyzed the influence of the three features on the experimental results
2. Compare the HOG extracted from the accumulated edge feature image and the original dance image
3. The recognition effect of the algorithm in this study on two dance datasets
4. Comparison between the proposed algorithm and the benchmark algorithm

The experimental results of the proposed algorithm and the benchmark algorithm on two dance datasets are analyzed and compared.

### 4.4. Results and Analysis

First, this study compares and analyzes HOG feature values extracted from feature membership images. The effect of action recognition in this study is different from the existing action, and the difference in the development is related to the extraction mode and calculation accuracy. The HOG advantages of the four groups of activities are given in Table 1.

The results in Table 1 clearly show the model's advantages in this study. The computational accuracy for follow step double flower combination model extraction results is 42.8%, 12% higher than the traditional model. For combination of cut and flower, the extraction results of this model were 40%, 20% higher than the conventional model. Towel flower combination model extraction results were 33.3%, 33.2% higher than the traditional model. Mosaic combination extracted 29.2%, 37% higher than the conventional model. The characteristic membership algorithm of the model in this study has significantly improved the calculation accuracy. It proves the validity of the model in this study. From the increase in accuracy, it is concluded that the recognition of the new model for subtle image differences is much higher than that of the traditional model.

Table 2 provides the experimental results of comparing the proposed method and the benchmark method in the four dance combinations of the FolkDance dataset.

The comparison of the commonly used centralized dance action recognition modes in the existing literature shows that the recognition rate of the new model in this study is higher than that of the traditional model. The highest accuracy is increased by 12.6%. The towel flower combination dance action selected in this study is very complex, and the accuracy is improved by 4.39%. The dance movement exists appropriately, and the accuracy is improved by 10.09. This result shows that the new fusion model in this study can not only improve the recognition accuracy in the fundamental recognition effect but also reflect the advantages of the particular action, complex action, and staggering occlusion action recognition.

## 5. Conclusions

This work mainly studies the selection and representation of features in dance movement recognition research and the fusion method of multimodal environmental monitoring data. The decisions are as follows:

1. Propose an effective method to extract the features of dance movements and divide dance movement videos equally. Accumulate the edge features of segmented videos. The edge features of all video images in each segment are added to one embodiment and extracted from the histogram features of the direction gradient. Aiming at the problem of heterogeneous feature fusion, three kinds of features are organically fused for dance action recognition through a multicore learning method, and the proposed fusion method can improve the dance recognition rate. Overall, the algorithm proposed in this study is more efficient than traditional methods.
2. In dance movement recognition, the direction gradient histogram feature, optical flow histogram feature, extracted audio element, and carry dance movement recognition are out by multifeature fusion. Aiming at the problem of heterogeneous feature fusion, organically fuse three kinds of features by a multicore learning method for dance movement recognition.
3. Make a FolkDance dataset. Develop a detailed dataset recording scheme. The Vicon motion capture system invites different dance majors to record dance videos according to dance group movement design. In the study for dance movement recognition research, the dataset concluded three people and four groups for 84 dance movement videos.

## Figures and Tables

**Figure 1:** HOG3D calculation process. (a) full descriptor (with 2x2x2 histogram cells) (b) histogram computation (over 2x2x2 sub-blocks) (c) gradient orientation quantization (d) mean gradient computation.

**Figure 2:** The various steps for computing HON4D.

**Figure 3:** Feature fusion process of multikernel learning.

**Figure 4:** Example frame of two-flower combination.

**Figure 5:** The sample frame of the mosaic combination.

**Figure 6:** Towel flower combination frame.

**Figure 7:** Sample frame of flower combination.

**Table 1:** Comparison of experimental results extracted from HOG.

Characteristics	Follow step double flower combination (%)	Combination of cut and flower (%)	Towel flower combination (%)	Mosaic combination (%)
HOG extraction in this study	42.8	40	33.3	29.2
Traditional HOG extraction [21]	38.1	33.3	25	21.3

**Table 2:** Comparison of experimental results.

Dance	Methods in this study (%)	Benchmarkmethod (%)
Follow step double flower combination	52.4	47.6 [22]
combination of cut and flower	53.3	60 [23]
Towel flower combination	50	47.9 [24]
Mosaic combination	45.8	41.6 [25]

## Data Availability

The data used to support the findings of this study are available from the corresponding author upon request.
